# Utility of the “BATS” Score in Predicting Choledocholithiasis in Patients With Gall Bladder Stones

**DOI:** 10.7759/cureus.42445

**Published:** 2023-07-25

**Authors:** Imdad Ali, Raja Taha Yaseen, Shoaib Ahmed Khan, Abbas Ali Tasneem, Syed Mudassir Laeeq, Hina Ismail, Nasir Hassan Luck

**Affiliations:** 1 Department of Hepatogastroenterology, Sindh Institute of Urology and Transplantation, Karachi, PAK; 2 Department of Gastroenterology, Sindh Institute of Urology and Transplantation, Karachi, PAK

**Keywords:** asge intermediate probability, endoscopic retrograde cholangiopancreatography (ercp), endoscopic ultrasound (eus), non-invasive, choledocholithiasis

## Abstract

Background and aim

The role of expensive, risky, and unnecessary endoscopic interventions can be avoided by the use of non-invasive tests to predict common bile duct (CBD) stones. Therefore, our aim was to identify non-invasive predictors of choledocholithiasis (CL) in patients and further to predict a model and assess its diagnostic accuracy in predicting CL.

Methods

This cross-sectional study was carried out from June 1, 2020, to December 31, 2021. Patients having gall bladder stones on percutaneous transabdominal sonography and fulfilling intermediate probability criteria of CL were enrolled. These patients then underwent radial endoscopic ultrasound (EUS) followed by endoscopic retrograde cholangiopancreatography (ERCP) for detecting CBD stones. Univariate logistic regression analysis, followed by multivariate logistic regression analysis, was performed to ascertain the independent predictors of CBD stone in patients with intermediate probability. A model was proposed, and the diagnostic accuracy was calculated at an optimal cutoff. The model was then internally validated in the patients with intermediate probability and was also compared with the pre-existing score.

Results

Out of 131 patients included in the study, CBD stone was noted in 85 (66%) and 88 (67.2%) patients on EUS and ERCP, respectively. On multivariate analysis, high serum bilirubin (>2 mg/dL) and alkaline phosphatase (200 IU) and dilated CBD (>6 mm) on transabdominal sonography at baseline were significant predictors of CBD stone in these patients. Using these variables, a scoring system (BATS score) was developed, which had an area under the receiver operating curve (AUROC) of 0.98 in predicting the presence of CBD stone with a sensitivity of 93.18%, a specificity of 76.74%, and a diagnostic accuracy of 87.79%. In the validation cohort, a BATS score of ≥5 had a diagnostic accuracy of 95.91% in predicting CL.

Conclusion

The BATS score showed excellent sensitivity and good diagnostic accuracy in predicting the CBD stone with excellent results on internal validation. However, external validation of our results is required to recommend this model on a larger scale.

## Introduction

One of the most commonly noticed problems in patients undergoing cholecystectomy for gall bladder stones or those presenting with signs and symptoms of biliary pancreatitis is choledocholithiasis (CL), comprising 5-10% and 18-33% of the cases, respectively [1-5]. Endoscopic retrograde cholangiopancreatography (ERCP) has currently been utilized as the gold standard technique for the management of CL. However, in the patients undergoing ERCP, the risk of certain complications such as post-ERCP pancreatitis, post-endoscopic sphincterotomy bleeding, cholangitis, and perforation can result in prolonged hospital stay, thus not only increasing the morbidity but also resulting in increased financial burden for the patient [6]. ERCP has shown cost-effectiveness only in the patients with the highest possibility of CL [7]. For the prediction of CL, 2010 ASGE guidelines proposed that the patients with a high probability of CL are the ones most likely to get benefit from endoscopic intervention. Secondly, the guidelines also forecasted the chances of the presence of CL in patients with suspected CL [8]. The guidelines further divided the patients into three categories. The first category included patients having a high possibility of common bile duct (CBD) stone, and the patients in this category should be managed by ERCP. The second category included patients with an intermediate probability of CL, and the patients in this category should undergo either endoscopic ultrasound (EUS) or MRCP for detecting CL. The size of the CBD stone has an influence on the utility of MRCP in detecting CBD stones as the sensitivity of MRCP decreases with a decrease in the size of the stone to <5 mm (67% vs 100%, if the size is ≥5 mm). On the contrary, when predicting CL of <5 mm, the sensitivity and diagnostic accuracy of EUS were far better than MRCP [9,10]. 

Previous studies have shown the utility of liver enzymes, like alkaline phosphatase (ALP) or gamma-glutamyl transpeptidase (GGT), individually in predicting CL [11,12]. Khan et al. [13] proposed a score named “AGT score” comprising ALP, GGT, and serum bilirubin for the prediction of CL with an excellent sensitivity of over 90% and a good diagnostic accuracy of 87%. However, this score was never validated, so it cannot be recommended at the moment.

Therefore, the main objective of our study was to identify the predictors of CL, to propose and internally validate the model, and to compare the proposed model with the previously existing score.

## Materials and methods

This cross-sectional study was carried out from June 1, 2021, to December 31, 2022, at the Department of Hepatogastroenterology, Sindh Institute of Urology and Transplantation (SIUT), Karachi, Pakistan, after the approval from the Ethical Review Committee (ERC). All the patients included have either dilated CBD (>6 mm) on percutaneous abdominal ultrasound or serum bilirubin between 1.8 and 4 mg/dL, along with any one of the following factors such as age greater than 55 years or deranged liver enzymes other than bilirubin, or history or presence of gallstone pancreatitis. EUS, followed by ERCP, was performed in all the included patients for detecting the presence or absence of CL.

IBM SPSS Statistics, version 22.0 (IBM Corp., Armonk, NY), was used for data entry and analysis. Mean + SD was used to express continuous variables, while frequencies and percentages were used to express categorical variables. Comparative analysis was done for continuous variables using the student t-test, and it was done for categorical variables using the chi-square test. Statistically significant factors on univariate analysis subsequently underwent multivariate analysis to identify independent predictors of CL. Using these variables, the “BATS score” was formulated and calculated for each patient.

The area under the receiver operating curve (AUROC) was obtained for the “BATS score.” The sensitivity, specificity, positive predictive value (PPV), negative predictive value (NPV), and diagnostic accuracy were obtained for the “BATS score” in the predicting CL. The BATS score was then internally validated, and its diagnostic accuracy was compared to that of the AGT score [13] in the studied population.

## Results

Out of 131 patients enrolled in the study, 106 (80.9%) were females. At baseline, abdominal pain was present in 127 (96.9%) patients, while pancreatitis was noted in 25 (19.1%) patients. At baseline, dilated CBD was present in 95 (72.5%) patients. On EUS, 85 (66%) patients had CL, while 88 (67.2%) patients on ERCP had CBD stone. On univariate analysis, female gender, presence of abdominal pain, dilated CBD at baseline, and high serum bilirubin, ALP, and GGT were significantly associated with the presence of CL (Tables 1, 2).

**Table 1:** Univariate analysis of the categorical variables in predicting choledocholithiasis in the studied population (n = 131) CBD, common bile duct; ERCP, endoscopic retrograde cholangiopancreatography

Characteristics		Stone on ERCP (n = 131)			p-value
		Yes		No	
Gender	Male	5	20		<0.001
	Female	83	23		
Abdominal pain	Present	88	39		0.004
	Absent	0	4		
Jaundice	Present	76	37		0.961
	Absent	12	6		
Dilated CBD	Present	72	23		0.001
	Absent	16	20		

**Table 2:** Univariate analysis of continuous variables included in the study (n = 131) TLC, total leucocyte count; AST, aspartate transaminase; ALT, alanine transaminase; GGT, gamma-glutamyl transpeptidase; ERCP, endoscopic retrograde cholangiopancreatography

Variables	Stone on ERCP	Mean ± SD (n = 131)	p-value
Age of the patient	Yes	53.4 ± 11.7	0.278
	No	50 ± 13.5	
Hemoglobin on admission (g/L)	Yes	12.9 ± 1.9	0.474
	No	12.7 ± 1.5	
TLC on admission	Yes	8.2 ± 2.3	0.584
	No	7.9 ± 1.2	
Platelets on admission	Yes	342 ± 77.9	0.760
	No	331 ± 80	
Creatinine on admission	Yes	0.85 ± 0.47	0.832
	No	0.9 ± 0.22	
Total bilirubin on admission	Yes	1.7 ± 0.9	0.043
	No	1.1 ± 0.4	
Alkaline phosphatase on admission	Yes	394 ± 103	≤0.001
	No	249.6 ± 143	
AST on admission	Yes	37.9 ± 29.9	0.797
	No	39 ± 32	
ALT on admission	Yes	62 ± 64	0.213
	No	48 ± 34	
GGT on admission	Yes	349 ± 171	0.049
	No	291 ± 248	
Serum amylase levels	Yes	137 ± 241	0.317
	No	235 ± 570	

On multivariate analysis, high serum bilirubin and ALP and the presence of dilated CBD on transabdominal sonography at baseline were independent predictors of CBD stone in these patients (Table 3).

**Table 3:** Multivariate analysis showing non-invasive independent predictors of CBD stone CBD, common bile duct; ALP, alkaline phosphatase; GGT, gamma-glutamyl transpeptidase

Variable	p-value	Odds ratio	CI (95%)	
			Lower limit	Upper limit
Female gender	0.089	0.951	0.898	1.008
Abdominal pain	0.143	0.542	0.432	0.691
Dilated CBD	<0.001	13.355	3.51	50.8
Total bilirubin	0.022	0.408	0.190	0.878
ALP	0.029	0.990	0.981	0.999
GGT	0.492	0.997	0.898	1.006

Using these variables, a scoring system (BATS score) (Table 4) was developed, which had an AUROC of 0.98 (p < 0.001) in predicting the presence of CL (Figure 1). In the “BATS” score, the scoring was done based on the odds ratio of the variable. Patients with dilated CBD had 13 times more odds of developing CBD stone compared to other variables; hence, it was given 3 points, while the other two variables were given two points each.

**Table 4:** Variables incorporated in the “BATS” score with allotted points (total points = 7) CBD, common bile duct; ERCP, endoscopic retrograde cholangiopancreatography

Variable		Stone on ERCP (n = 131)		Points allotted (total = 7)
		Present	Absent	
Bilirubin >2 mg/dL	Yes	79	14	2
	No	14	45	
Alkaline phosphatase >200 IU	Yes	93	22	2
	No	0	37	
Dilated CBD on transabdominal ultrasonography	Yes	74	8	3
	No	19	51	

**Figure 1:** AUROC for the “BATS” score was 0.98 (p < 0.001) AUROC, area under the receiver operating curve

A cutoff value of a BATS score of ≥5 demonstrated a sensitivity of 93.18%, a specificity of 76.74%, a PPV of 89.13%, an NPV of 84.62%, and a diagnostic accuracy of 87.79% in predicting CBD stone in patients with intermediate probability (Table 5).

**Table 5:** Sensitivity, specificity, PPV, NPV, and diagnostic accuracy of the “BATS” score in predicting choledocholithiasis PPV, positive predictive value; NPV, negative predictive value

Statistics	BATS score >5	95% CI
Sensitivity	93.18%	81.34% to 98.57%
Specificity	76.74%	57.74% to 91.38%
PPV	89.13%	77.06% to 93.29%
NPV	84.62%	69.74% to 95.51%
Accuracy	87.8%	77.30% to 94.04%

The sample size of the validation cohort was 346. Out of them, 274 (79.2%) were females. Abdominal pain was noted in 330 (95.4%) patients, while jaundice was noted in 50 (14.5%) patients. On percutaneous ultrasound, CBD was dilated in 243 (70.2%) patients (Table 6).

**Table 6:** The baseline characteristics of the validation cohort (N = 346) CBD, common bile duct

Characteristics		N (%)
Gender	Males	72 (20.1)
	Females	274 (79.2)
Abdominal pain	Present	330 (95.4)
	Absent	16 (4.6)
Jaundice	Present	50 (14.5)
	Absent	296 (85.5)
Dilated CBD	Present	243 (70.2)
	Absent	103 (29.8)
Age of the patient (years)		47.4 + 13.1
Total bilirubin on admission (mg/dL)		1.7 + 0.89
Alkaline phosphatase on admission (IU)		339.6 + 134

A BATS score of ≥5 had a sensitivity of 97.25%, a specificity of 93.55%, a PPV of 96.36%, an NPV of 95.08%, and a diagnostic accuracy of 95.91% in predicting CL. When compared with the AGT score, the BATS score had higher diagnostic accuracy along with excellent sensitivity, specificity, PPV, and NPV in predicting CL (Table 7).

**Table 7:** Sensitivity, specificity, PPV, NPV, and diagnostic accuracy of “BATS” and “AGT” scores in the validation cohort for the prediction of choledocholithiasis (N = 346) PPV, positive predictive value; NPV, negative predictive value

Statistics	BATS score >5	95% CI	AGT score >463	95% CI
Sensitivity	97.25%	94.11% to 98.98%	92.66%	88.35% to 95.75%
Specificity	93.55%	87.68% to 97.17%	73.39%	64.70% to 80.92%
PPV	96.36%	93.13% to 98.11%	85.96%	82.01% to 89.15%
NPV	95.08%	89.77% to 97.71%	85.05%	77.81% to 90.22%
Accuracy	95.91%	93.23% to 97.74%	85.67%	81.50% to 89.21%

## Discussion

Previously, the guidelines showed a lack of accuracy for the suspected CL. EUS is a technique that is proven to be an exceptional means for the management of various diseases in the field of hepato-pancreato-biliary system. Many endoscopists prefer radial EUS because of the clear and extensive visualization of biliary ducts [14,15]. Previously, studies have revealed an excellent diagnostic accuracy of EUS with an excellent sensitivity for detecting CL of <5 mm with no impact on the stone size on its accuracy [16].

Previous studies have shown the utility of liver enzymes, like ALP or GGT, individually in predicting CL [11,12]. Khan et al. [13] previously proposed an AGT score in 71 patients, showing a sensitivity of 93.18%, a specificity of 77.78%, and a diagnostic accuracy of 87.3% in predicting CL. Similarly, Kadah et al. [17] proposed that dilated CBD on ultrasound, increased age, and GGT were independent predictors of CBD stone and also developed a model using these scores, which had an AUROC of 0.73. Tunruttanakul et al. [18] proposed a model for predicting CL, comprising advanced age, dilated CBD on percutaneous ultrasound, higher serum bilirubin, and ALP levels with an AUROC of 0.80. However, in our study, serum tests that included parameters of liver function such as total bilirubin and ALP, along with dilated CBD (>6 mm) on percutaneous ultrasound, were independent predictors of CL.

Therefore, using these parameters, we proposed a model named “BATS” score for patients with suspected CL, which showed a significant association with CL and also had a higher AUROC than the previous studies, i.e., 0.98. A “BATS” score of ≥5 had an excellent diagnostic accuracy of 87.8% and excellent sensitivity and specificity in predicting CL.

 In comparison with the AGT score, the BATS score had excellent sensitivity, PPV, NPV, and diagnostic accuracy in predicting CBD stone in patients with intermediate probability.

Certain limitations to our study included the lesser sample size, and the external validation of our model was not carried out.

There were several strengths that can be attributed to our study. Firstly, it was the cross-sectional nature of the study. Secondly, the proposition of a non-invasive cost-effective score for the prediction of CL was one of the major strengths of this study. Third, the diagnostic accuracy of the BATS score was compared with the other coexisting score. Lastly, the internal validation of the score was performed.

## Conclusions

Compared to the previously existing models, the “BATS” score performed significantly better for predicting CL in patients with suspected CBD stone, falling in the intermediate probability of CL with excellent sensitivity, specificity, and diagnostic accuracy. However, for the further recommendation of this score on a larger scale, multicentric studies with large sample sizes are required.
